# Ultrasound Calibration for Dual-Armed Surgical Navigation System

**DOI:** 10.1155/2022/3362495

**Published:** 2022-02-16

**Authors:** Kuan-Ju Wang, Chieh-Hsiao Chen, Chun-Yi Lo, Hung-Hsin Lin, Jia-Jin Jason Chen

**Affiliations:** ^1^Department of Biomedical Engineering, National Cheng Kung University, Tainan, Taiwan; ^2^Brain Navi Biotechnology Co. Ltd, Zhubei, Hsinchu Country, Taiwan; ^3^China Medical University Beigang Hospital, Yunlin County, Taiwan

## Abstract

Ultrasound (US) imaging system is widely used in robotic systems for precision positioning in clinical applications. The US calibration is critical to minimize the difference of spatial coordinates between instruments, for minimally invasive surgery (MIS) in navigation systems. In this study, we propose a dual robotic arm system that combines US imaging with one arm for path planning and monitoring and accurate positioning with the other arm for instrument placement via the preplanning procedures. A phantom with N-wire and N-wedge was designed for US calibration. The US calibration showed a mean error of 0.76 mm; the mean dual-arm calibration error is 0.31 mm. The positioning error of the system was verified with a mean error of 1.48 mm. In addition, we used two abdominal phantoms with computed tomography scan validation, with an averaged position error of 1.867 ± 0.436 mm and an orientation error of 2.190 ± 0.764°. The proposed system is aimed to perform clinical operations, such as abdominal MIS, with real-time image monitoring of the organ tissues and instrument positions, which meet the requirements for medical application.

## 1. Introduction

Surgical navigation is a critical system making the existing treatment procedures more accurate or approaching new possible procedures [1]. The procedures of minimally invasive surgery (MIS) require the targeted insertion of instruments for diagnostic or therapeutic purposes, such as biopsy, surgery, and radiotherapy [2]. The advanced image navigation system is assisted to provide patients with high-precision radiotherapy or surgical treatment and improvement of treatment effectiveness. Ultrasound (US) imaging is widely used in the clinic with its high temporal resolution, noninvasion, and high controllability. The US-guided navigation system can provide real-time monitoring, nidus targeting, and more accurate results [3]. Several integrated US-guided robotic systems have been proposed for precision positioning in clinical applications. For example, a mounted needle insertion with a US-guided robot was designed for percutaneous puncture which can improve the positioning and orientation accuracies than free-hand puncture [4]. In the integrated system, the US arm calibration is essential to minimize the difference of spatial coordinates between US images and instruments.

For the calibration between the US image and robotic arm with instruments, the localization of identified objects from the US image to system coordinate is based on the transducer position. The localization data of the robotic arm and the US transducer including position and orientation are required [5]. Trackers or mechanical arms are commonly used for collecting such data for calibration. Many tracker-based systems utilizing various tracking technologies have been proposed, providing the most maneuverability combined with US real-time imaging property [6]. In contrast, the mechanic arm can locate the positioning more accurately and has the ability to focus on a specific area or target by fixing the location with a US transducer [7]. To perform the US calibration, the phantom is commonly used to obtain the transformation from tracked coordinates to image coordinates. Various types of phantom models have been demonstrated, such as single or multiple point targets, cross-wire, 2D shape alignment, Z-fiducial (or N-fiducial), and wall phantoms [8–10]. These phantoms are designed with specific features to determine the world coordinates for the tracking system, and therefore, the objects observed in the US image can be located. However, for a US-guided navigation system, the treatment procedures are highly dependent on the operators [11]. Many free-hand US systems or US-instrument integrated system have been proposed to track the operations, but the localization and the operations with these systems depend on the medical experts' experiences that largely affect the outcome of the treatment [8].

To minimize the invasion and maximize the outcome of the treatment, in this paper, we propose a dual robotic arm system for MIS. The system combines US image acquisition with one arm for path planning and the accurate positioning with the other arm for instrument placement via the preplanning path. The calibration for the US image and the two arms was based on an in-house designed multiwire and N-wedge phantom. Finally, it is important to analyze not only positioning errors but also the orientation of the proposed system, and therefore, the system was verified by using a verification phantom and two abdominal phantoms for positioning and orientation accuracy test. The designed system is aimed to perform clinical operations with real-time image monitoring of the organ tissues and instrument positions.

The organization of this paper is listed as follows: (1) The first part introduces the background, motivation, and the aim of this study. (2) The second part describes the materials and methods of the dual robotic arm system in detail, including the instruments, spatial transformation, calibration, and integration methods. The calibration and verification methods with the designed experiments are introduced. (3) The third part analyses the results of calibration experiments for US image, US to arm transformation, dual-arm calibration, and the results of the verification for the US imaging-guided dual-arm system. The accuracy of the system is described by the spatial deviation and orientation. (4) Finally, we summarize the system and the results of the experiments and point out the importance of the system for clinical requirements.

## 2. Materials and Methods

The procedures include four phases: the hardware calibration, the USarm operation, the TLarm operation, and the system validation (Figure 1). The calibration procedures included the calibration between US image and arm, dual robotic arm calibration, the operations of two arms (the robotic arm with US transducer, USarm, and the robotic arm with tool, TLarm) with US image, and the validation. The dual robotic arms were calibrated by recording a set of the positions of robotic arms, and transformation between both was calculated. The coordinate system transformation from the US image to two arms was applied from hardware calibration. The system was validated by the difference between the target point and the standard stylus point. The symbols for the calibration system and spatial information used in this study are listed in Table 1.

### 2.1. Hardware Configuration

The architecture of the system is comprised of four items, including two six-axis robotic arms, an ultrasound imaging system, and the control system. In this study, the calibration between US image and arm is performed by one robotic arm to acquire the US image of the phantom. The spatial information from the US image was identified based on the manufacturer and experimental data. The distance features between objects from the US image were used to compare the designed values for transformation calculation. With a combination of the dual-arm and image-arm spatial transformations, the compartments of the system were aligned and then validated by measuring the positions of two robotic arms by assigning the points from the US image. The calibrated system is designed for imaging, planning, and operating the preplanned procedures for surgical navigation. Two collaborative robotic arms of Universal robots UR5e (Universal Robots, Odense, Denmark) with 6 degrees of freedom were used in this system, which provide flexible control components for system setup. The movement repeatability of UR5e is ±0.03 mm, and the working range is within 850 mm. One arm was designed to hold the US transducer and the other one was designed to hold the instruments, which were fixed on the trolley. The arm which held the US transducer was defined as USarm, and the other which equipped the tools (e g., stylus or instruments) was defined as TLarm. The US system of BenQ T3300 (BenQ Corporation, Taipei, Taiwan) was used, which is equipped with the transducer of C62 B sector-type linear array, 128 channels of the phased array, and the frequency of 2.0 ∼ 6.0 MHz. The output image resolution of the capture card is 1920*∗*1080. A calibration phantom was designed in combination with N-wire and N-wedge. The wires provide precise spatial positions, and the planes have geometric features. It can improve the system accuracy from image processing. The sheet features are used to confirm the spatial positioning and to reduce errors caused by ultrasound image resolution. In addition, we designed three feature points {*p*_*o*_, *p*_*x*_, *p*_*y*_}_*P*_ on the calibration phantom surface, which were used for the robotic arm to get the coordinates on the phantom. The calibration phantom was placed in a tank filled with water. The calibration phantom with the designed features is shown in Figure 2. For system verification, a homemade pyramid-shaped phantom and two abdominal phantoms, CIRS-057A and CIRS-071B (Computerized Imaging Reference Systems, Inc. (CIRS), Norfolk, USA), were used. The pyramid sharp points were designed for ultrasound imaging detection; the abdominal phantoms included several features such as organs or tumors that were used as target points. A coordinate-measuring machine (CMM), HEXAGON Romer absolute arm 7312 (HEXAGON, Stockholm, Sweden) with point repeatability of ±0.014 mm, was used for measuring three-dimensional coordinates, providing the surface shape and coordinates of the object with a contact probe. CMM was fixed on the same platform with two robots and was able to probe the coordinate of the tip of the robots and the markers of phantoms. The symbols for the coordinate system and transformation between each coordinate system in the system are listed in Table 1.

### 2.2. Rigid-Body Transformation

A rigid body refers to an object whose shape and size remain unchanged during movement and after being subjected to a force, and the relative position of the internal points of the object (e g., arms, instruments, or phantom) does not change. Rigid transformation of the plane preserves length, involving reflection, translation, and rotation. In this study, the least-squares approximation method was used to transform the spatial coordinates of the two known sets of corresponding points. In order to transform an arbitrary set of points **P**_*I*_ and **P**_*P*_ from the **W**_*I*_ to **W**_*P*_, the optimized translation *T* and rotation *R* need to be calculated. The minimum of the sum of squares was used for optimization, as follows:

(1) $$\begin{array}{c} \text{min}\sum \left(R*P_{I}+T\right)-P_{P}^{2}. \end{array}$$

The control points **P**_*I*_ and **P**_*P*_ were known as corresponding points, and the optimal solution for transformation could be calculated based on a closed-form solution and quaternion method [12, 13]. The cross-covariance matrix can be calculated by the following equation:

(2) $$\begin{array}{c} \sum_{\text{IP}}=\frac{1}{N}\sum_{i=1}^{N}\left[\left(P_{I}-{\overset{⟶}{\mu }}_{I}\right){\left(P_{P}-{\overset{⟶}{\mu }}_{P}\right)}^{T}\right], \end{array}$$

where ${\overset{⟶}{\mu }}_{I}$ and ${\overset{⟶}{\mu }}_{P}$ are the center of mass. The cyclic components of the antisymmetric matrix *A*_*ij*_=(Σ_IP_ − Σ_IP_^*T*^)_*ij*_ were used to form the column vector Δ=[*A*_23_  *A*_31_  *A*_12_]^*T*^, and this vector was then used to form the symmetric 4×4 matrix *Q*(Σ_IS_) as

(3) $$\begin{array}{c} Q\left(\Sigma_{\text{IP}}\right)=\left[\begin{array}{cc} tr\left(\Sigma_{\text{IP}}\right) & \Delta^{T}\\ \Delta & \Sigma_{\text{IP}}-\Sigma_{\text{IP}}^{T}-tr\left(\Sigma_{\text{IP}}\right)I_{3} \end{array}\right], \end{array}$$

where *I*_3_ is the 3×3 identity matrix. The unit eigenvector ${\vec{q}}_{v}={\left[q_{0}\;q_{1}\;q_{2}\;q_{3}\right]}^{t}$ corresponding to the maximum eigenvalue of the matrix *Q*(Σ_IP_) was selected as the optimal rotation. The rotation matrix is described as follows:

(4) $$\begin{array}{c} R=\left[\begin{array}{ccc} q_{0}^{2}+q_{1}^{2}-q_{2}^{2}-q_{3}^{2} & 2\left(q_{1}q_{2}-q_{0}q_{3}\right) & q_{1}q_{3}+q_{0}q_{2}\\ 2\left(q_{1}q_{2}+q_{0}q_{3}\right) & q_{0}^{2}+q_{2}^{2}-q_{1}^{2}-q_{3}^{2} & 2\left(q_{2}q_{3}-q_{0}q_{1}\right)\\ 2\left(q_{1}q_{3}-q_{0}q_{2}\right) & 2\left(q_{2}q_{3}-q_{0}q_{1}\right) & q_{0}^{2}+q_{3}^{2}-q_{1}^{2}-q_{2}^{2} \end{array}\right]. \end{array}$$

The optimal translation vector *T* is given by

(5) $$\begin{array}{c} T={\overset{⟶}{\mu }}_{P}-R{\overset{⟶}{\mu }}_{I}. \end{array}$$

### 2.3. Ultrasound Image Calibration

US image was used to guide the robotic arm for instrument positioning. The object coordinates from the ultrasound image were aligned to the coordinate system of the robotic arm. The coordinate transformation of US image to USarm was defined as **T**_*I*_^USarm^.  Figure 3 illustrates the transformations during ultrasound image calibration. The transformation **T**_*I*_^USarm^ was calculated by the following equation:

(6) $$\begin{array}{c} T_{I}^{\text{USarm}}=T_{\mathrm{USarm}}^{P}*T_{P}^{I}. \end{array}$$

At the first step, we calculated the transformation between the **USarm** and the phantom (**T**_**USarm**_^*P*^). The phantom coordinate system was preidentified by CMM. We operated the robotic arm with a standard stylus to each feature position of the phantom and recorded the robotic coordinates {*p*_*o*_, *p*_*x*_, *p*_*y*_}_*T*Larm_. The unit vectors ${\vec{v}}_{1}$ and ${\vec{v}}_{2}$ were calculated by

(7) $$\begin{array}{c} {\vec{v}}_{1}=\left\{\frac{P_{1}-P_{0}}{\left|P_{1}-P_{0}\right|}\right\},\\ {\vec{v}}_{2}=\left\{\frac{P_{2}-P_{0}}{\left|P_{2}-P_{0}\right|}\right\}. \end{array}$$

The eigenvectors ${\vec{v}}_{x}$, ${\vec{v}}_{y}$, and ${\vec{v}}_{z}$ were calculated by the vectors ${\vec{v}}_{1}$ and ${\vec{v}}_{2}$, which were used to define the transformation *T*_**USarm**_^Phantom^. The equations are expressed as follows:

(8) $$\begin{array}{c} {\vec{v}}_{x}={\vec{v}}_{y}\times {\vec{v}}_{z},\\ {\vec{v}}_{z}={\vec{v}}_{1}\times {\vec{v}}_{2},\\ {\vec{v}}_{y}={\vec{v}}_{z}\times {\vec{v}}_{1},\\ T_{\mathrm{USarm}}^{\text{Phantom}}=\left[\begin{array}{cccc} {\vec{v}}_{x\left(x\right)} & {\vec{v}}_{y\left(x\right)} & {\vec{v}}_{z\left(x\right)} & p_{0\left(x\right)}\\ {\vec{v}}_{x\left(y\right)} & {\vec{v}}_{y\left(y\right)} & {\vec{v}}_{z\left(y\right)} & p_{0\left(y\right)}\\ {\vec{v}}_{x\left(z\right)} & {\vec{v}}_{y\left(z\right)} & {\vec{v}}_{z\left(z\right)} & p_{0\left(z\right)}\\ 0 & 0 & 0 & 1 \end{array}\right]. \end{array}$$

In the second step, we established the transformation between the ultrasound image and the calibration phantom (**T**_*P*_^*I*^). The ultrasound transducer was used to scan the calibration phantom perpendicular to the base from above. Image denoising was performed by Gaussian binomial filter [14]. The edges of the objects in the US image were detected by Canny edge detection, and the circles and lines were segmented [15, 16]. The circles on the image were corresponding to the lines of the calibration phantom, and the lines on the image were corresponding to the planes of the calibration phantom. After feature detection, six-point set *P*_*I*_={*p*_1_, *p*_2_,…,*p*_6_}_*I*_ and three-line set **L**_*I*_={*l*_1_, *l*_2_, *l*_3_}_*I*_ on the images were obtained. From **P**_*I*_ and **L**_*I*_, the feature point set from the image **P**_*I*_={*p*_1_, *p*_2_,…,*p*_12_}_*I*_ was identified, which was the corresponding phantom point set **P**_*P*_={*p*_1_, *p*_2_,…,*p*_12_}_*P*_, as shown in Figure 2(a). The image pixel size **T**_scale_ was calculated by **P**_*I*_ and **P**_*P*_, and **S**_*x*_ and **S**_*y*_ represented the scale of the *X*-axis and *Y*-axis in the US image by following equations:

(9) $$\begin{array}{c} T_{\text{scale}}=\left[\begin{array}{cccc} S_{x} & 0 & 0 & 0\\ 0 & S_{y} & 0 & 0\\ 0 & 0 & 0 & 0\\ 0 & 0 & 0 & 1 \end{array}\right],\\ S_{x}=\frac{1}{3}\left(\frac{{\left\{\overset{\leftarrow }{p_{1}p_{2}}\right\}}_{I}}{{\left\{\overset{\leftarrow }{p_{1}p_{2}}\right\}}_{p}}+\frac{{\left\{\overset{\leftarrow }{p_{3}p_{4}}\right\}}_{I}}{{\left\{\overset{\leftarrow }{p_{3}p_{4}}\right\}}_{p}}+\frac{{\left\{\overset{\leftarrow }{p_{5}p_{6}}\right\}}_{I}}{{\left\{\overset{\leftarrow }{p_{5}p_{6}}\right\}}_{p}}\right),\\ S_{Y}=\frac{1}{4}\left(\frac{{\left\{\overset{\leftarrow }{p_{1}p_{3}}\right\}}_{I}}{{\left\{\overset{\leftarrow }{p_{1}p_{3}}\right\}}_{p}}+\frac{{\left\{\overset{\leftarrow }{p_{3}p_{5}}\right\}}_{I}}{{\left\{\overset{\leftarrow }{p_{3}p_{5}}\right\}}_{p}}+\frac{{\left\{\overset{\leftarrow }{p_{2}p_{4}}\right\}}_{I}}{{\left\{\overset{\leftarrow }{p_{2}p_{4}}\right\}}_{p}}+\frac{{\left\{\overset{\leftarrow }{p_{4}p_{6}}\right\}}_{I}}{{\left\{\overset{\leftarrow }{p_{4}p_{6}}\right\}}_{p}}\right). \end{array}$$

**P**_*P*_ is only defined with the *X-* and *Y*-axis values. In order to obtain the scan position in the three-dimensional space, the *Z*-axis value, denoted as **P**_*P*−*z*_, is needed to be calculated. Based on the design of the calibration phantom, the coordinates *m*_1_, *m*_2_, *m*_3_ in the coordinate system of the calibration phantom are shown in Figure 2(b). The points {*p*_10_}_*p*_, *P*_*P*_{*p*_12_}_*p*_, *m*_1_, *m*_2_, and *m*_3_ were used to calculate **P**_*P*−*z*_ based on similar triangles, as shown in Figure 2(b). The equation is as follows:

(10) $$\begin{array}{c} P_{\mathrm{P-Z}}=\frac{{\left\{\overset{\leftarrow }{m_{1}m_{3}}\right\}}_{P}}{{\left\{\overset{\leftarrow }{m_{2}m_{3}}\right\}}_{P}}*{\left\{\overset{\leftarrow }{p_{10}p_{12}}\right\}}_{P}. \end{array}$$

The transformation **T**_*P*_^*I*^ between the ultrasound image and the calibration phantom was obtained from the image featured point set **P**_*I*_ and corresponding phantom point set **P**_*P*_. Finally, the coordinate systems of the US image and **USarm** were aligned by the transformation **T**_*I*_^USarm^=**T**_**USarm**_^*P*^*∗ ***T**_*P*_^*I*^.

### 2.4. Dual Robotic Arm Calibration

In this section, we describe the dual robotic arm calibration method and verification by CMM. To integrate the dual robotic arm workspace for collaborative working, the transformation *T*_USarm_^TLarm^ between both the robotic arms needed to be obtained. Two robotic arms, CMM, and the phantom were mounted on the stable platform and not moved during the measurement procedure. Before measuring the position of the dual robotic arm, each robotic arm's tool center point (TCP) was defined at the original flange. We predefined a set of the robotic arm's TCP position *P*_def_={*p*, *p*_2_, *p*_3_,…,*p*_*n*_}_def_ and operated the robotic arm to the target pose for each robot arm. This defined pose was within a specific area that CMM was able to measure it. The CMM was used to locate the featured mechanism on the robotic arm's flange and record the three-dimensional coordinate in each predefined position. The set of measured points was defined as *P*_USarm_={*p*, *p*_2_, *p*_3_,…,*p*_*n*_}_USarm_ and *P*_TLarm_={*p*_1_, *p*_2_, *p*_3_,…,*p*_*n*_}_TLarm_. According to the rigid transformation method stated above, we were able to compute the transformation **T**_USarm_^CMM^ and **T**_TLarm_^CMM^ between the robotic arm and the CMM coordinate system by two known sets of corresponding points. The transformation *T*_USarm_^TLarm^ between two robotic arms was defined as follows:

(11) $$\begin{array}{c} T_{\text{USarm}}^{\text{TLarm}}=T_{\text{TLarm}}^{\text{CMM}-1}\;*T_{\text{USarm}}^{\text{CMM}}. \end{array}$$

### 2.5. System Integration

Figure 4 illustrates the system architecture with two arms, the US transducer, the standard stylus, and the phantom. The positioning of the proposed dual robotic arm system was aligned from the US image coordinate system (**W**_*I*_), two arms coordinate systems (**W**_USarm_ and **W**_TLarm_), calibration phantom coordinate system (**W**_*P*_), and stylus coordinate system (**W**_*s*_). The coordinate transformations of US image to USarm (**T**_*I*_^USarm^), USarm to TLarm (**T**_USarm_^TLarm^), and TLarm to standard stylus (**T**_TLarm_^*S*^) were computed for the alignment of coordinate systems. The equation of the transformation between the target points {*p*_target_} in the coordinate systems of US image and stylus from **W**_*I*_ to **W**_*s*_ is described as

(12) $$\begin{array}{c} {\left\{p_{\text{target}}\right\}}_{S}=T_{\text{TLarm}}^{S}*T_{\text{USarm}}^{\text{TLarm}}*T_{I}^{\text{USarm}}*{\left\{p_{\text{target}}\right\}}_{I}. \end{array}$$

### 2.6. System Verification

The verification of the dual robotic arm system was tested by various phantoms in two phases. First, the homemade pyramid-shaped calibration phantom was used (Figure 5). The shape point of the pyramid was set as the target point. The TLarm with a stylus was driven to the target point by setting an appropriate path. The CMM was used to measure the coordinates of the target point and the stylus tip for distance errors. The procedure was repeated 30 times. Second, the RFA experiments with abdominal phantoms were performed to simulate the ablation in surgery (Figure 6). The TLarm with radiofrequency ablation (RFA) needle (CelonProSurge 150-T40) was driven to the target point by setting an appropriate path from the skin surface via US image-guided planning (Figure 6(a)) and 6(b)). The CT scans of two abdominal phantoms were performed before and after the needle insertion experiments (Figure 6(c)). The CT images were analyzed to extract the needle positioning and orientation errors for verification (Figure 6(d)). The verification procedure with abdominal phantoms was repeated 14 times, 7 times for each. The RFA needle was implemented on TLarm for precise positioning. Two models of standard image guide abdominal biopsy phantom. These simplified abdominal phantoms are suitable for training and demonstrating image-guided needle biopsy navigation tools or procedures that require a constant visual reference for needle placement.

## 3. Results

### 3.1. US Image Calibration

Based on the N-wedge phantom proposed by Lin et al. (2018) [17], we designed a phantom with six wires and the planes for US calibration. The scanned features in the US image are shown in Figure 7. The pixel size of the US image was 0.16 ± 0.001 mm of the *x*-axis and 0.16 ± 0.002 mm of the y-axis, representing the width and the depth, respectively.  Figure 7(a) is the original US image obtained by scanning the calibration model. After image processing and feature extraction (Figures 7(b) and 7(c)), US image with 12 feature points was identified (Figure 7(d)). From these featured points, US image calibration is to calculate transformation between US images and the calibration model. To verify the accuracy of the ultrasound image calibration method, we tested a set of independent verification experiments. After US calibration via calibration phantom, the ultrasound probe has performed the scan of the verification phantom and identified the feature points  {*p*_target_}_*I*_ on the ultrasound image. The feature position of the phantom was measured by CMM and denoted as {*p*_phantom_}_CMM_.

The top feature of the pyramid was selected for verification (Figure 5). We transformed {*p*_target_}_*I*_ and {*p*_phantom_}_CMM_ to **W**_USarm_ and calculated the deviation. The verification was performed with the pyramid-shaped verification model. The registration error of the tip point between the US image and the verification model was calculated (Figure 8(a)). The mean *x*-axis, *y*-axis, and *z*-axis errors were 0.475 ± 0.464 mm, 0.193 ± 0.289 mm, and 0.311 ± 0.312 mm, respectively. Our US calibration showed a mean error of 0.759 ± 0.296 mm. The results of the US calibration were highly influenced by US image quality and resolution. Besides, the image artifact of phantom reflection, US beamwidth, and focal zone were the major factors for error accumulation in image processing.

### 3.2. Dual-Arm Calibration

To verify the repeatability of the dual robotic arm after calibration, we first set three groups of position movements for USarm. We set the same coordinate movement and multiply the movement by **T**_USarm_^TLarm^ for TLarm. The transformations between two robotic arms included translation and rotation. CMM was used to measure these positions of two robotic arms. The distribution of error distance is shown in Figure 8(b). The mean errors of the three verifications calibration error were 0.2848 ± 0.043 mm, 0.331 ± 0.061 mm, and 0.328 ± 0.053 mm, respectively. The max errors in the three verifications are 0.413 mm, 0.531 mm, and 0.406 mm, respectively. The mean of the three independent experiments calibration error is 0.314 ± 0.052 mm.

### 3.3. System Accuracy

#### 3.3.1. Experimental Analysis with the Verification Phantom

A standard stylus was used to perform the positioning for system verification. Target position {*p*_target_}_*I*_ was transformed to robot base coordinate system {*p*_target_}_*S*_ by predefined transformation (1). The robotic arm TLarm with the stylus was driven to the target pose and recorded the tool position {*p*_target_}_CMM_ by CMM. The position deviations between {*p*_phantom_}_CMM_ and {*p*_target_}_CMM_ are shown in Figure 8(c). The mean system error in 10 experiments was 1.477 ± 0.405 mm. Our system indicated that the error distribution of the *x*-axis was relatively large, which might be the unstable positioning caused by the US beamwidth in the US calibration. Our results showed that the accuracy of US positioning can still be maintained at the same level compared to other studies [8, 18, 19].

#### 3.3.2. Experimental Analysis of the RFA Insertion with Abdominal Phantoms

The results of positioning and orientation error in 7 experiments for CIRS-057A were 1.828 ± 0.240 mm and 2.239 ± 0.947 degrees (Figure 9(a)) and in 7 experiments for CIRS-071B were 1.907 ± 0.593 mm and 2.141 ± 0.600 degrees (Figure 9(b)). The results of positioning and orientation error of these 14 experiments were 1.867 ± 0.436 mm and 2.190 ± 0.764°. In the postoperative CT images, the RFA needle showed some deviation during the process of entering the phantom. It might be attributed to two potential factors, the rigidity of the probe and the insertion angle. The rigidity of the needle might be led to the deviation caused by penetrating the tissues of the phantom while the needle might be bent by the surface elasticity. The positioning error could have resulted from the length of the needle and the elastic characteristic parameter of its materials. In addition, as shown in Figure 9(c), the positioning error would be larger as the insertion depth increased due to the orientation error. Taken together, depending on the scenarios of surgery, the characteristics of instruments would be considered, and the trend estimation provides the reference for depth optimization while performing surgery. The proposed system showed the precise positioning and orientation by testing the error compared by the RFA practice and planning path with abdominal phantoms. The dual robotic arm with the US image-guided system is aimed to perform clinical operations, such as abdominal MIS.

## 4. Conclusion

In this study, the operation of the system was designed for surgical procedures. We focused on the accuracy of the overall system and established a high accuracy robotic arm surgical guided system. The pros and cons of each hardware calibration and registration would greatly affect the accuracy of the proposed system. The dual robotic arm integration, US image spatial calibration, and system integration are critical factors for highly precise surgical robot system design. However, the collaborative robots UR5e were used for system implementation, but a certificated robot for use in surgery is needed in the next stage. In this work, the system is simply integrated with the coordinating transformation; however, the treatment is highly dependent on the accuracy of the positioning to perform the presurgical planning strategy. Our current results of the hardware calibration and system can provide the precision positioning to meet the clinical requirement for MIS. Further improvement for the clinical environment and workflow as well as adapting it to patient and operation environment for clinical applicability is needed.

## Figures and Tables

**Figure 1:** The flowchart of the calibration system. The procedures include four phases: the hardware calibration, the USarm operation, the TLarm operation, and the system validation. The hardware calibration included: (a) The transformation between the US image and USarm was calculated via the US image and the designed geometry of the calibration phantom. (b) The transformation between USarm and TLarm was obtained by pointing a set of points on one comment target. For procedures (1) to (4), the coordinate system transformation from the US image to two arms was applied from hardware calibration (a, b). (1) The calibration phantom was scanned by USarm. (2) The coordinate system transformation was applied from US image to USarm. (3) The base-to-base transformation was applied from USarm to TLarm. (4) The TLarm with the standard stylus was moved to the target position via US image planned path from (1). (5) The system was validated by the difference between the target point and the standard stylus point.

**Figure 2:** The calibration phantom. (a) Calibration phantom and feature points that could be detected by the US image. The red lines on the plan indicate the scan projection from the US image. (b) The side view of the calibration phantom. The dotted line represents the slice of the US image, which is perpendicular to the phantom. The feature points of the calibration phantom are designed to calculate the position of the slice.

**Figure 3:** Transformations during ultrasound image calibration.

**Figure 4:** The coordinate systems and the relationships between US image, arms, and the object (phantom). The transformations of US image to USarm (**T**_*I*_^USarm^), USarm to TLarm (**T**_USarm_^TLarm^), and TLarm to standard stylus (**T**_TLarm_^*S*^) were computed for the dual robotic arm positioning system guided by the ultrasound image. The target points in the coordinate system of US image {**p**_**target**_}_**I**_ and in the coordinate system of stylus {**p**_**target**_}_*S*_ should be aligned after transformation.

**Figure 5:** The pyramid-shaped verification phantom. The 3D structure model (a) and the US image (b).

**Figure 6:** The RFA insertion with US image-guided experiment. (a) US image-guided RFA insertion. (b) The needle was visualized by 3D reconstruction on the CT image with US image slice (as shown in bottom left). The green point shows the needle position. (c) The CT scan after insertion. (d) The reconstructed planning path and the RFA needle from the CT image.

**Figure 7:** Ultrasound image processing and feature detection. (a) Original ultrasound image. (b) The edge detection for feature circle and lines. (c) The extension of the detected circle and lines for feature points based on the design of the calibration phantom. (d) The detection of the feature points corresponding to the calibration phantom.

**Figure 8:** The system verification with the positioning errors. (a) The ultrasound image calibration results, including the *x*-axis, *y*-axis, *z*-axis, and distance errors. (b) Dual robotic arm calibration results in three independent experiments. (c) The system verification with image-guided stylus pointing, including the *x*-axis, *y*-axis, *z*-axis, and distance errors.

**Figure 9:** The experimental analysis of the RFA insertion with two abdominal phantoms (CIRS-057A and CIRS-071B). (a) The distance of positioning errors of RFA needle insertion between the planning path and the RFA needle. (b) The orientation error of RFA insertion between the planning path and the RFA needle. (c) The calculated trend of the positioning error based on the orientation error with insertion depth.

**Table 1:** The symbols for the coordinate system and transformation.

Symbol	Description
**U** **S** **a** **r** **m**	Robotic arm with ultrasound transducer
**T** **L** **a** **r** **m**	Robotic arm with tool
**W**_**U** **S** **a** **r** **m**_	USarm base coordinate system
**W**_**T** **L** **a** **r** **m**_	TLarm base coordinate system
**W**_**I**_	Ultrasound image coordinate system
**W**_**P**_	Calibration phantom coordinate system
**W**_**s**_	Standard stylus coordinate system
{**p**_**target**_}_**I**_	Target in ultrasound image coordinate system
{**p**_**target**_}_**S**_	Target in standard stylus coordinate system
**T**_**I**_^**U** **S** **a** **r** **m**^	Transformation from ultrasound image to USarm
**T**_**U** **S** **a** **r** **m**_^**T** **L** **a** **r** **m**^	Transformation from USarm to TLarm
**T**_**T** **L** **a** **r** **m**_^**S**^	Transformation from robotic TLarm to standard stylus
**T**_**scale**_	Ultrasound image pixel size

## Data Availability

The data used to support the findings of this study are available from the corresponding author upon request.
